RETRACTED

# KANO Model-Enabled Performance Evaluation of Urban Public Sports Services

**DOI:** 10.1155/2022/1749616

**Published:** 2022-06-07

**Authors:** Yang Liu, Wei Wei

**Affiliations:** ^1^Department of Physical Education, College of General Education, Guangdong University of Science & Technology, Dongguan 523083, China; ^2^School of Physical Education and Sports Science, South China Normal University, Guangzhou 510630, China

## Abstract

Starting from the goal of overall equalization of basic public services by 2035 as proposed in the report of the 19th Party Congress, firstly the research history of the equalization of public sports services in China is analyzed in stages, and a solid theoretical foundation is laid for the construction of the evaluation index system. Secondly, the performance evaluation system of urban public sports services, which is based on KANO model, is constructed by combining the current development status of public sports services in China. Additionally, fuzzy KANO model is used to analyze and categorize the collected indicators and establish a user-oriented evaluation index system. Finally, an empirical study was conducted on a region using the evaluation system, and the results showed that the degree of equalization of public sports services in the region was achieved to a high degree and was basically close to reaching the target requirement of equalization.

## 1. Introduction

From the Fifth Plenary Session of the 16th Central Committee of the Communist Party of China, which for the first time proposed the equalization of basic public services, to the 18th National Congress of the Communist Party of China, which focused on the goal of comprehensively improving people's living standards and emphasized the overall realization of the equalization of basic public services, and finally to the report of the 19th National Congress of the Communist Party of China, which emphasized the overall realization of the equalization of basic public services, by 2035, the equalization of public services should be largely completed, demonstrating that the fulfillment of equalization has been a central goal of the Party and the government from the beginning of their existence. Consequently, the establishment of a scientific and effective evaluation index system for the equalization of basic public services has become one of the measures proposed by the central government to carry out the important spirit of the 19th Party Congress report, and it has also become one of the core index systems used to measure high-quality economic and social development in the country. It is an important part of public services to conduct research on the fundamental concepts and evaluation dimensions of the degree of equalization, which is also a positive response to the current major theoretical needs of the central decision-making department and is conducive to the realization of equalization in basic public services throughout the country. The degree's assessment index system is being built at the time of this writing [1–5].

RETRACTED

In order to understand the customer demand and its relationship to the customer satisfaction, the Japanese researcher Kano Noriaki developed the KANO model, which divides the influential elements of the customer satisfaction into four categories. Because of the model's ongoing refinement and promotion, the KANO model is currently widely used throughout the world. In many sectors, fulfilling client demands is at the heart of what we do. Some researchers used the fuzzy KANO questionnaire to analyze and develop an optimization model for product functional requirements in order to address the issue of insufficient consideration of the autocorrelation relationship between functional requirements in traditional quality function development. Users' expectations of product satisfaction and product cost are efficiently reconciled through the process of gathering personalized requirements [6, 7]. Some researchers have developed approaches for designing analytical KANO models, which are intended to alleviate the difficulties that can arise when categorizing criteria using KANO models. Obtaining an objective classification of quality characteristics is the goal. According to some researchers, the Kano two-dimensional quality model is used to examine consumers' satisfaction with different service quality aspects using the Kano questionnaire and then to identify the most important service quality factors to focus on. According to the above research findings, the KANO model is a relatively accurate and efficient research tool when analyzing user demand-centered evaluation problems; however, most scholars use the KANO model to conduct simple user surveys, demand analysis, or index classification, among other things. The five classification standards built into the KANO model are used to screen, classify, and categorize the indicators that are now in general usage in the field of public sports service quality evaluation as described in this paper. Integration is followed by the development of an evaluation index system that is dominated by user requirements and geared toward quality assurance.

In order to objectively evaluate the quality of urban public sports services, in addition to a reasonable index system, a rigorous evaluation technique is also required in order to conduct an objective evaluation. Some researchers begin with industrial design as the starting point for product design evaluation and then analyze and summarize the evaluation methods used throughout the development process. They also introduce information to describe the uncertainty of the index weight and then develop a design scheme based on the principle of maximum abstraction to achieve the best results. Some researchers employ the TOPSIS approach or the VIKOR method to assess the degree to which the various perceptual dimensions between the alternatives and the needs of the users are aligned. Following a review of the literature, it was discovered that the majority of assessment methods for urban public sports services are based on a handful of standard multi-criteria evaluation approaches. However, while it has some usefulness in solving the product design evaluation problem that is oriented on user needs, the technique described above has also the following two shortcomings: the multicriteria decision-making methods TOPSIS and VIKOR are both multicriteria decision-making methods with extreme solutions as reference solutions. Although alternatives that are infinitely close to the optimal solution can be selected, it is expected that the solution that best meets the preferences and expectations of users within an acceptable cost range will be found. In contrast, if users' subjective optimal expectations are chosen as the decision-making aim, there will inevitability be a problem in that users' subjective optimal expectations will not be achievable due to the restrictions of practical conditions. (2) In the process of product design, not just technology, materials, and components are considered, but those are considered as well [8–10]. This, the user's volatility should be taken into consideration during the evaluation process. They are not only numerous, but also impossible to measure, and they are basically a vague concept in and of themselves. The evaluation process itself involves judgment and subjectivity, which means that the results of the evaluation will inevitably be more ambiguous than the process itself.

RETRACTED

In order to address these issues, we have developed a hesitant fuzzy sets-enabled KANO model (FKANO) to improve the standardization phase that is required to increase the application of method. With reference to the historical development of equalization in the nations, this research creates a set of evaluation index systems to measure the actualization of equalization in public sports services from the perspective of academic evolution. Complete achievement of the equality of fundamental public sports services serves as both a theoretical reference and a practical guide in both theory and practice.

The rest of the paper is organized as follows.

In next section, the research process of the equalization of basic public sports services in our country is reported along with supportive literature contents. In Section 3, the performance evaluation of urban public sports service based on FKANO model is presented along with other models. Results of the proposed fuzzy-enabled KANO model are compared with the state-of-the-art approaches as shown in the results section. Finally, summarized contents are provided to conclude the paper.

## 2. The Research Process of the Equalization of Basic Public Sports Services in My Country

The adoption of the leadership model gives a fresh perspective and a solid platform for the EHRQA's work, clarifies the fundamental responsibilities of the human resources department, and establishes a solid base for enterprise development. Meanwhile, it serves as a solid foundation for the company's personnel recruiting, job assignment, employee training and development, promotion and reward performance, and other activities, and it heralds the beginning of a new chapter in the growth of human resources [11].

### 2.1. Institutional Establishment Stage: 2005–2011

The Fifth Plenary Session of the 16th Central Committee of the Communist Party of China adopted the “Proposal of the Central Committee of the Communist Party of China on Formulating the Eleventh Five-Year Plan for National Economic and Social Development” on October 11, 2005, marking the first time the equalization of basic public services has been implemented at the national level. The proposal was adopted by the Central Committee of the Communist Party of China on October 11, 2005. The method had been established and had been well explained. Since then, the debate over the equalization of public services across a wide range of social sectors has continued to rage on the Internet. The equalization research of public sports service has begun to expand rapidly as a significant field of public service. It is also becoming a more important field of public service. For example, a scholar, working in education sector, draws the essence of equalization of public services. He points out that equalization of public sports services means that people from different classes and regions can benefit equally from public sports resources. Additionally, he proposes to develop public sports service infrastructure projects in underdeveloped areas, among other things. The nonequalization of basic public services, according to some other scholars, is now the primary constraint on the development of a moderately prosperous society on an all-around basis. It is necessary to further clarify the three connotations of equalization in public sports services, namely, the equalization of choice rights, the equalization of participation opportunities, and the equalization of service results. From the standpoint of fairness, citizens' sports rights serve as the primary foundation for the provision of public sports services, and the dual structure of urban and rural separation serves as the primary reason for the inequality of citizens' sports rights and the nonequalization of public sports service provision [12–14].

RETRACTED

The following are the characteristics of this phase of the study:

1. Equalization research in other domains serves as a valuable source of information: this period's research on equalization of public services was heavily impacted by the household registration system, which is necessary due to historical reasons relating to the dual structure of urban and rural areas in my nation at the time of its inception. It is being implemented a social welfare system, which includes compulsory schooling, a collective pension, and public medical care, in both the realms of medical care and education. This historical cause has directly contributed to the fact that fundamental public services are mostly provided to urban people, whereas farmers are unable to take advantage of the same basic public services as urban residents. Secondly, time factor is another important aspect that is hard to the farmer to follow a specific schedule as his service structure has a very different set of requirements. In addition, because sports were a marginal public service at the time, its study material was primarily concerned with the basic public service ideals of “urban-rural division” and “city-based operation.” It can be shown that there were a considerable number of urban-rural and interregional public sports services that were equal in terms of equity in the CNKI database. There are various findings of the research.
2. Examine the equality of public sports services from the standpoint of fairness and justice, as well as other considerations: the Communist Party of China's 17th National Congress declared in its report in 2007 that the starting point should be to accelerate socialist construction that is centered on improving people's livelihoods, and to strive to promote social and economic development, coordinate and improve people's livelihood issues, and promote social fairness and justice as a starting point. We have observed that the government has begun to follow those ideologies, which are people-oriented and fair. Likewise, equalization of public services has created a new situation: the basic medical and health systems in both urban and rural areas have been fully established. Free compulsory education system in both urban and rural areas has been fully realized. Basic pension insurance system in both urban and rural areas has been fully implemented. In the realm of public sports services, it is also proposed to defend the fundamental sports rights of farmers and to investigate the possibility of equalizing the provision of public sports services in urban and rural areas. Although this equalization is done through a vast number of financial subsidies and tax incentives, as well as other economic ways to obtain fair results, the government's operation incurs significant economic expenses as a result of this equalization [15, 16].

RETRACTED

### 2.2. Theoretical Exploration Stage: 2012–2016

On July 11, 2012, the State Council issued the “Twelfth Five-Year Plan for the National Basic Public Service System,” which listed public sports services as an important content separately. It also clarified from the top that sports belonged to the category of public services and that public sports received the same services as other public sports, among other things. In-depth research of chemistry has established the groundwork for a theoretical framework. From the perspectives of welfare economics and resource allocation theory, some scholars have discussed the critical role played by human, financial, material, and other resources in the equalization of public sports services, and they have proposed that the equitable distribution of sports resources requires reasonable institutional constraints in order to ensure that supply and demand are equal in public sports. The subject of who will supply public sports services, as well as what and how they will supply public sports services, has been raised by several academics, who have provided theoretical support for the implementation of equalization in public sports services from the perspective of supply. Other researchers argue that the theoretical foundation for the equalization of public sports services comprises not only economic concepts, but also traditional theories from the domains of management, sociology, and political science, among other things. Existing problems were identified, and a realistic basis for promoting the equalization of public sports services was systematically analyzed from six perspectives: national cognition, economic foundation, public sports facilities, sports social organizations, volunteer services, and laws and regulations. It was concluded that China should begin at a lower level and work its way up from there. It is steadily increased until it equalizes with the higher standard, at which point it becomes equalized with the higher standard [17–23].

RETRACTED

The following characteristics distinguish this phase of study:

1. The research perspective gradually shifts from the demand side to the supply side: in contrast to the previous stage, which began with demand, the study conducted in this stage is primarily concerned with the provision of public sports services. First and foremost, from the standpoint of supply security, it is recognized that the national financial system is the most significant factor in achieving the equalization of public service delivery. The book then begins with the supply standard for public sports service and goes on to explain the standardization of public sports service from a variety of viewpoints throughout the book. However, because of the wide range of social preferences, it is only possible to conclude that standards are generally dynamic in nature. As far as supply is concerned, most of it comes from the government's acquisition of public sports services, but the supply process has been hampered in numerous ways and has failed to achieve true supply equality in the market. For supply content, as people's sports demands continue to grow, new outdoor ventures such as rock climbing and automobile camping are becoming increasingly popular with the general population. Ice and snow events have also begun to penetrate the public's field of vision, particularly since Beijing and Zhangjiakou were awarded the right to host the 2022 Winter Olympics in 2015 [24, 25].
2. Have a more in-depth understanding of the concept of equalization: because of its historical trajectory, it is clear that new China has always sought equality as an ideal and as a goal in all areas of life: politics and economics; social and cultural life. It is because of the pursuit of this ideal of equality that, in the realm of public sports services, the low-level average state is being followed blindly, notwithstanding recent improvements. Real equalization of public sports services, on the other hand, has reached a mature stage, and the level of public sports services not only achieves relative equality between different regions, between urban and rural areas and between individual residents, but also actively participates in social forces in terms of supply, resulting in a multiparty system. For the equalization of sports services in the public sector, participation, standardization, flexibility, and control of an effective management system are required. More mature equalization approaches in foreign countries include the following: the government guarantees equalization of bottom line income, and social forces provide high-quality public services in order to achieve the linkage effect of government finance and social capital, thereby achieving relative equalization [26].

RETRACTED

### 2.3. Practical Operation Stage: 2017 to Present

This study argues that this stage corresponds to the operation stage of refined practice, based on the logical reasoning of goal achievement and the theoretical investigation conducted in the previous stage. Furthermore, the “Thirteenth Plan for Promoting the Equalization of Basic Public Services,” which was released in the 13th Five-Year Plan, focuses on promoting the equalization of the construction of the basic public service system and proposes the policy goal of promoting the overall realization of the equalization of basic public services. A specific fulcrum has been identified for the evaluation of the level of development of equalization of public sports services in the United States. In some study, it has been claimed that the equalization of public sports services is comprised of distinct goals at different phases such as overarching objectives, process objectives, and result objectives. Some academics believe that, by examining public sports services in developed countries abroad, it is proposed that, in order to achieve true equalization of public sports services, it is necessary to actively guide the participation of citizens and social forces, in order to enable social capital or organizations to provide high-quality and personalized public sports services, and to establish public sports services. The pattern of joint investment of private capital and public financing is protected by the diversification guarantee. In addition, using research methods such as the literature method and logical analysis method, other academics have elaborated on the meaning of the term “equalization of public sports services” and developed an assessment index system for the term “equalization of public sports services.” It is planned to investigate the equalization of public sports services in the form of index data in order to make recommendations. Some researchers use the city of Shenzhen as an example for conducting an empirical study on the equalization development level of public sports services, and they feel that there are still nonequalization phenomena in many parts of the city's sports services [27, 28].

The following are the main characteristics of this phase of research:

1. The goal of equalization of public sports services is clearly defined: the 13th Five-Year Plan, when compared to previous discussions on the equalization of public services, expresses a clear commitment to achieving a realistic goal of equalization of basic public services by 2020. It also outlines requirements and points out the direction for the development of equalization of public sports services. On the macro level, the government must continue to make financial investments in the development of a public sports service system, as well as improve the procedural and legal framework for government procurement of services. A medium-term goal should be achieved through the diversification of supply subjects, the diversification of supply contents, and the platformization of supply routes, among other initiatives. It is vital, from a micro perspective, to establish scientific and diverse evaluation indicators and implement data-based performance evaluation in order to accomplish success. In contrast, the equalization of public sports services is a people's livelihood project about which the government has been concerned for a long time, and it involves a wide variety of and difficult interactions, which the government has been concerned about for a long time. More research is needed to determine how to attain the goal of equalization from macro, meso, and micro viewpoints, among others.
2. The participation of social forces results in a greater variety of evaluation indicators being developed: practices in other parts of the world and in other areas of people's livelihood have demonstrated that encouraging the government to purchase public sports services from social forces is an important way to increase sports consumption demand while also enriching the supply of public services. It is also extremely important for the realization of equalization of public sports services in China. In terms of policy, the General Office of the State Council issued the “Guiding Opinions on Government Purchase of Services from Social Forces” in 2013, and the provision of public sports services by social forces has emerged as an important means of achieving equalization. In terms of practice, the State General Administration of Sports and the People's Government of Zhejiang Province signed the “Framework Agreement of the State Sports General Administration and the People's Government of Zhejiang Province” in September 2017, which established that Wenzhou City, in the province, has been designated as the country's first pilot city for the organization of sports by social forces. As a result, given the increasingly important role played by social forces in the provision of urban public sports services, it is imperative to establish an evaluation index system for the equalization of urban public sports services that incorporates the majority of the supply of social forces in order to serve as a theoretical reference and theoretical foundation for the achievement of equalization goals in other cities, a guidance on how to do things.

RETRACTED

## 3. Performance Evaluation of Urban Public Sports Service Based on FKANO Model

In the decades since its introduction in the 1980s, the KANO two-dimensional model has grown to become one of the most widely used quality models among management practitioners and researchers across a wide range of industries. Its primary purpose is to illustrate and determine the quality attributes of research objectives. This model does away with the idea that product impact on customer satisfaction is strictly linear, allows for the classification of specific attributes that may affect customer satisfaction, and acknowledges that the relationship between customer demand fulfillment and customer satisfaction is nonlinear. The many sorts of requirements are classified into the following categories:

1. Charismatic quality (A): if there is enough of these elements in the product, customer happiness will be considerably boosted as a result of the presence of this element; if there are inadequate or no such elements in the product, consumers will not be satisfied. As a result, the customer is dissatisfied with the product.
2. One-dimensional quality (O): the adequacy or lack of such quality components will have an impact on a user's pleasure with a product. As an essential quality aspect, increasing the sufficiency of this element can lead to an improvement in customer satisfaction, and the converse is true, a condition characterized by a linear drop in consumer satisfaction.
3. Required quality (M): this type of quality factor is the critical component that customers believe must be included in the product. If this type of aspect is not properly reflected in the product, client happiness will soon deteriorate as a result of the inability to deliver the essential performance. Contrary to this, no matter how much the adequacy of such parts is increased, the resulting influence on user satisfaction is only marginally higher.
4. Indifferent quality (I): users' pleasure does not alter when such elements are changed, indicating that they are not significant to them.
5. Quality (R): if the performance of this type of quality element is sufficient, user satisfaction will fall, and if the performance of this type of quality element is insufficient, it will lead to an increase in user satisfaction. It is possible that the customer's contentment with the specific quality of the product or service will be questioned. As illustrated in Figure 1, there is a wide range of preferences for mass qualities.

After collecting user questionnaires, we classified the categories of criteria and indicators expected by users and eliminated the indicators that did not meet their expectations, resulting in the development of a quality evaluation index system for product design schemes that are oriented toward user expectations (see Table 1). Because users have diverse attitudes and priorities when it comes to different types of quality factors, this study establishes the criteria weights and index weights in the KANO model based on the classification types of quality factors. However, because the product features of different items differ, a uniform standard cannot be established, and the standard must be altered in accordance with the real product and customer attitude in question. The detailed indicator settings are the same as those in [12].

RETRACTED

Developing an evaluation method that can not only adapt to its index system but meet its decision-making goals along with user's needs, the index system is based on the division of KANO quality factors, and it serves as the foundation for the quality evaluation of product design schemes. This is a critical step. Following an in-depth examination of various research findings, it is discovered that the multiobjective and multicriteria characteristics of product design scheme quality evaluation determine that this problem is a typical multicriteria decision-making problem with multiple objectives and multiple criteria. Furthermore, the uncertainty of user expectations, as well as the limits of decision-making specialists, is also present in this situation. It establishes an atmosphere of ambiguity for the criterion. In order to address the issues raised above, this work develops an FKANO evaluation model that is applicable to the situation. Evaluation index system of basic public sports services is shown in Table 1.

Let *X* be a given set, and let *M*={*u*_1_, *u*_2_,…, *u*_*n*_} be the *N* membership functions of the given set, and then the hesitant fuzzy set about the membership function *M*, that is, *H*_*M*_, is defined as

(1) $$\begin{array}{c} H_{M}=\left\{\langle x,h_{M}\left(x\right)\rangle |x\in X\right\}, \end{array}$$

where *h*_*M*_(*x*)=*U*_*u*∈*M*_{*u*(*x*)} is a set whose value range is located on [0,1], indicating that the element *x* of *X* in the set belongs to several possible membership degrees of the set *H*_*M*_.

For the convenience of expression, the whole hesitant fuzzy set on the finite universe *X* is denoted as HFS(*x*), and *h*_*A*_(*x*) is called the hesitant fuzzy element of *A*.

For any three hesitant fuzzy elements *h*_1_, *h*_2_, and *h*_3_, their algorithm is as follows:

(2) $$\begin{array}{c} h_{1}\cap h_{2}=H\left\{\min\left(\alpha_{1},\alpha_{2}\right)|\alpha_{1}\in h_{1},\alpha_{2}\in h_{2}\right\},\\ h_{1}\cup h_{2}=H\left\{\max\left(\alpha_{1},\alpha_{2}\right)|\alpha_{1}\in h_{1},\alpha_{2}\in h_{2}\right\},\\ \theta h=H\left\{1-{\left(1-\alpha \right)}^{\theta }|\alpha \in h,\theta >0\right\},\\ h^{\theta }=H\left\{\alpha^{\theta }|\alpha \in h,\theta >0\right\},\\ h^{c}=H\left\{1-\alpha |\alpha \in h\right\},\\ h_{1}⊕h_{2}=H\left\{\left(\alpha_{1}+\alpha_{2}-\alpha_{1}\alpha_{2}\right)|\alpha_{1}\in h_{1},\alpha_{2}\in h_{2}\right\},\\ h_{1}⊗h_{2}=H\left\{\alpha_{1}\alpha_{2}|\alpha_{1}\in h_{1},\alpha_{2}\in h_{2}\right\}. \end{array}$$

Let *h*_*a*_, *h*_*b*_ be any two hesitant fuzzy elements, and then the distance formula between the hesitant fuzzy elements *h*_*a*_, *h*_*b*_ is calculated as

(3) $$\begin{array}{c} d\left(h_{a},h_{b}\right)=1-\frac{1}{2}\#h_{a}\sqrt{\prod_{r_{a}\in h_{a}}\left(1-\#h_{b}\right)\left|r_{a}-r_{b}\right|}-\frac{1}{2}\#h_{b}\sqrt{\prod_{r_{b}\in h_{b}}\left(1-\#h_{a}\right)\left|r_{a}-r_{b}\right|}, \end{array}$$

where #*h*_*a*_ represents the number of elements in the hesitant fuzzy element *h*_*a*_, and #*h*_*b*_ represents the number of elements in the hesitant fuzzy element *h*_*b*_.

RETRACTED

Let *h*(*x*) be the fuzzy unit, and then *s*(*h*(*x*))=1/#*h*(*x*)∑_*α*∈*h*(*x*)_*α* is the score function of *h*(*x*), where #*h*(*x*) represents the element number contained in *h*(*x*).

Given two hesitant fuzzy elements *h*_*a*_ and *h*_*b*_, if *s*(*h*_*a*_) > *s*(*h*_*b*_), then *h*_*a*_ > *h*_*b*_; if *s*(*h*_*a*_)=*s*(*h*_*b*_), then *h*_*a*_=*h*_*b*_.

## 4. Results

Beijing is chosen as the city for empirical research in this study, and the FKANO model is used to undertake a full evaluation of it using the newly constructed index system. At various stages throughout the entire evaluation process, different types of groups, such as experts and scholars working in the field of sports research in Beijing, relevant leaders from sports departments, social sports instructors, and sports enthusiasts, are brought together to ensure the scientific and rational nature of the results. First, the weights of different evaluation findings from various evaluators are calculated, and then the final evaluation conclusion is calculated by conducting a full study of FKANO and other relevant data. For the purpose of determining the degree to which the equalization of public sports services has been achieved, this study divides the evaluation results into five categories: fully realized, nearly realized, generally realized, partially achieved, and not achieved at all, referred to as *V* = variational equalization of public sports services (completely realized, nearly realized, generally realized, not realized, and not realized at all). Without a doubt, the grade number is an ambiguous numerical figure that is inconvenient for intuitive evaluation and that fluctuates within a specific range. The % system is, therefore, commonly employed in actual operation to indicate the evaluation criterion for each grade level. The equalization interval should be 60–69 points, the median value is 65 points, and the equalization will not be realized at all. The near-achievement interval should be 80–89 points, the middle value is 85 points, the general realization interval should be 70–79 points, the middle value is 75 points, and the unrealized interval should be 60–69 points, and the median value is 65 points. Let us evaluate the value range between 50 and 60 points for the time being (a value of less than 50 points signals a major concern), with the median value being around 55 points.

RETRACTED

The participants in the single-factor evaluation were 40 direct recipients of public sports services in Beijing (general sports enthusiasts), and the effective evaluation level was divided into five categories: fully realized, nearly realized, generally realized, not realized, and not realized at all. The participants in the single-factor evaluation were 40 direct recipients of public sports services in Beijing (general sports enthusiasts). The following is the relationship matrix for the FKANO model evaluation that was obtained:

(4) $$\begin{array}{c} R=\left[\begin{array}{cccc} \begin{array}{c} 0.135\\ 0.166 \end{array} & \begin{array}{c} 0.551\\ 0.388 \end{array} & \begin{array}{c} 0.423\\ 0.345 \end{array} & \begin{array}{c} \begin{array}{cc} 0.011 & 0.000 \end{array}\\ \begin{array}{cc} 0.113 & 0.000 \end{array} \end{array}\\ 0.786 & 0.456 & 0.345 & \begin{array}{cc} 0.015 & 0.000 \end{array}\\ 0.366 & 0.493 & 0.132 & \begin{array}{cc} 0.016 & 0.000 \end{array}\\ \begin{array}{c} 0.242\\ 0.283 \end{array} & \begin{array}{c} 0.412\\ 0.577 \end{array} & \begin{array}{c} 0.219\\ 0.126 \end{array} & \begin{array}{cc} \begin{array}{c} 0.055\\ 0.026 \end{array} & \begin{array}{c} 0.000\\ 0.000 \end{array} \end{array} \end{array}\right]. \end{array}$$

According to the aforementioned matrix, the second item has a pretty high monetary worth. The idea of maximum membership is used to determine if sports enthusiasts in Hangzhou, Zhejiang Province, believe that the equalization level of public sports services has been achieved or is close to being achieved, according to preliminary findings.

It is a difficult task to assess the progress made toward the goal of equalization of fundamental public sports services provided by all organizations. Even if it is merely from the perspective of sports enthusiasts, the outcome will be considerably distorted due to the point of view and other factors. During the actual evaluation process, this study included four types of evaluation groups, including local experts and scholars, administrative leaders, sports instructors, and sports enthusiasts, in a thorough manner, as well as 0.2. Finally, the same procedure was used to get a single-factor comprehensive evaluation of the various evaluation groups using the same evaluation groups as before. The findings are presented in Table 1.

(5) $$\begin{array}{c} S=D\times V\\ =82.36. \end{array}$$

Through a multifactor examination, it has been determined that Beijing has achieved 82.36 percent of its goal of equalizing the provision of fundamental public sports services to all citizens.

RETRACTED

Further, based on the urban public sports service level calculated by experts, the FKANO model proposed in this paper is compared with the KANO model and the TOPSIS model. The comparison cities are Beijing, Shanghai, and Hangzhou. The result is shown below.

From Figures 2–4, it can be found that the estimated value of the FKANO model is the closest to the predicted value of the experts.

## 5. Conclusion

In this paper, we have examined stage equalization of public sports services in our nation, which provides a sound theoretical foundation for the effective development of an assessment index system. The FKANO model and hesitant fuzzy sets are integrated into the sports service performance evaluation system. In addition, the fuzzy KANO model is used to analyze and classify the indicators that have been collected, as well as to develop a user-oriented assessment index system for cities. Finally, utilizing the evaluation system provided in this research, an empirical investigation is carried out in a specific area, which confirms the superiority of the FKANO assessment method over other existing state-of-the-art evaluation methods.

## Figures and Tables

**Figure 1:** Structure of KANO.

**Figure 2:** Comparison of the different models in Beijing.

**Figure 3:** Comparison of the different models in Shanghai.

**Figure 4:** Comparison of the different models in Hangzhou.

**Table 1:** Evaluation index system of basic public sports services.

Overall system level	Criterion layer
The degree of equalization of basic public sports services	Supply resources
	Supply subject
	Supply quality
	Supply efficiency
	Demand level
	Outcome level

## Data Availability

The data used to support the findings of this study are available from the corresponding author upon request.
